RETRACTED

# A Chaotic Neural Network Model for English Machine Translation Based on Big Data Analysis

**DOI:** 10.1155/2021/3274326

**Published:** 2021-07-02

**Authors:** Qianyu Cao, Hanmei Hao

**Affiliations:** ^1^School of Foreign Languages, Chengdu University of Information Technology, Chengdu 610036, China; ^2^Chengdu Angke Technologies Co., Ltd., Chengdu 610000, China

## Abstract

In this paper, the chaotic neural network model of big data analysis is used to conduct in-depth analysis and research on the English translation. Firstly, under the guidance of the translation strategy of text type theory, the translation generated by the machine translation system is edited after translation, and then professionals specializing in computer and translation are invited to confirm the translation. After that, the errors in the translations generated by the machine translation system are classified based on the Double Quantum Filter-Muttahida Quami Movement (DQF-MQM) error type classification framework. Due to the characteristics of the source text as an informative academic text, long and difficult sentences, passive voice, and terminology translation are the main causes of machine translation errors. In view of the rigorous logic of the source text and the fixed language steps, this research proposes corresponding post-translation editing strategies for each type of error. It is suggested that translators should maintain the logic of the source text by converting implicit connections into explicit connections, maintain the academic accuracy of the source text by adding subjects and adjusting the word order to deal with the passive voice, and deal with semitechnical terms by appropriately selecting word meanings in postediting. The errors of machine translation in computer science and technology text abstracts are systematically categorized, and the corresponding post-translation editing strategies are proposed to provide reference suggestions for translators in this field, to improve the quality of machine translation in this field.

## 1. Introduction

With the rapid development of Internet-related technology, increased websites have opened user reviews for a certain event or a certain type of product and because of the huge number of Internet users, each type of website will generate a huge amount of data for each type of event every day, and these data in various formats and of different lengths will have great commercial and social value when they are formed in scale [1]. For example, analysing certain types of products of a certain store can help merchants discover the information that users are mainly concerned about when buying products, thus improving the quality of service and generating commercial value; for customers, customers generally consider the cost performance of products when buying and selling, and in the case of the same cost performance, the evaluation of other customers who have already purchased plays a crucial role in deciding whether users themselves buy; for shopping platforms, analysing the evaluation of all users is crucial to discovering the shortcomings of platform management; analysing the evaluation of these Internet users is crucial to discovering the shortcomings of platform management. For shopping platforms, analysing all users' comments is crucial to find out the shortcomings of platform management; analysing these netizens' comments can keep abreast of the public opinion guidance, social climate, and people's outlook and values. However, in the face of such a huge amount of data, how to extract useful information from them has become a hot topic of concern in recent years. One of the subtasks of text sentiment classification is to extract useful information from the huge amount of data to provide a reference value for product sales, public opinion analysis, and policymaking [2]. Text sentiment classification has become a hot research topic in recent years.

RETRACTED

In today's explosive growth of data and information, we have access to a huge amount of data and information every day [3]. To make this information help modern society develop better and faster, we need to discover the laws contained in this information and make accurate predictions, so data mining and deep learning technologies are born. Shopping malls will arrange products regularly according to customers' buying habits, advertisers will put out push ads according to consumers' habits and preferences, and media will put out news and current events that readers like and care more about according to their reading habits. Deep learning technology has influenced our life in every aspect, and we can feel a lot of convenience in it [4]. Similarly, deep learning can also help teachers and students to manage and interact more conveniently in educational scenarios. For example, the current cloud classroom technology can bring knowledge to students outside of the classroom and make education more popular by getting rid of the traditional education confined to the classroom. Deep learning technologies are also bringing changes to the education evaluation system, and classroom emotion is one of the directions [5]. In this paper, we demonstrate the design of Sirius, the open end-to-end IPA web service software that allows users to ask questions via voice and pictures, and it responds in natural language. We then use this workload to investigate four implications in the design space of a future accelerator-based server architecture that includes central processing units (CPUs), general-purpose processors (GPUs), multiple core throughput coprocessors, and field-programmable gate arrays (FPGAs). To study the future server design of Sirius, we decompose Sirius into a suite with eight detection programs inside (Sirius Suite), including Sirius' compute-intensive bottlenecks [6]. We put the Sirius Suite on a series of gas pedal platforms and used its performance and power trade-offs on these platforms to analyse the total cost of ownership (TCO) of different server design points [7]. We found that gas pedals are pivotal to the future stability of IPA services. Our results show that GPU-accelerated servers and FPGA-accelerated servers reduce query latency by an average of 8.5x and 15x, respectively. For a given throughput, GPU-accelerated servers and field-programmable gate array (FPGA)-accelerated servers reduce TCO by a factor of 2.3 and 1.3, respectively, across data centers.

RETRACTED

We demonstrate a method that synthesizes sensible acoustic effects at an interactive rate in a large dynamic environment containing multiple sound sources. Our concept combines listener-based backward ray tracing with sound source clustering on board and hybrid audio rendering for complex scenes. We give a new algorithm for dynamic post-reverberation that performs higher-order ray tracing in the listener on spherical sound sources. We achieve sublinear scaling with the number of sources by aggregating distant sources and considering their relative intelligibility. We also describe a hybrid convolution-based audio rendering technique that can process hundreds of thousands of sound paths at interactive rates. We demonstrate the performance of this algorithm in indoor-outdoor scenes with up to 200 sound sources. In practice, our algorithm can compute over 50 reflection instructions at an interactive rate on a multicore PC, and we also observe that it is up to 5 times faster than previous geometric sound propagation algorithms.

## 2. Current Status of Research

Bansal et al. proposed a lexicon-based approach to extract sentiment from text, designing the Sentiment Tendency Calculator (SO-CAL) that uses a lexicon labeled with sentiment tendencies (polarity and intensity) as a basis for judgment and fuses negative lexicons to assign corresponding sentiment labels to the text [8]. Chen et al. believed that the text should contain adjectives or adverbs [9]. García-Ródenas et al. consider adjectives or adverbs contained in the text as an important basis for determining the emotional polarity of the text, and by calculating the mutual information difference with the specified words separately, the average emotional tendency value of the text is obtained [10]. The main way to build sentiment lexicon is to expand the required sentiment lexicon according to certain rules based on existing sentiment lexicon, which can be constructed manually, heuristic algorithms, and machine-learning algorithms [11]. And most of the learning algorithms based on sentiment dictionaries use propagation algorithms to estimate the sentiment value of each word; that is, the similarity between words is calculated using the results of syntactic analysis, contextual information, and linguistic information provided by sentiment dictionaries [12]. Supervised learning includes both classification and regression, and as the representative of supervised learning, the research of classification methods occupies a pivotal position in the whole development of machine learning, especially in the fields of artificial intelligence technology and big data analysis technology, which have exploded in the last decade. Most of the traditional classification methods and their derivatives take the physical attributes of the target, such as distance, colour, and similarity, as sample features, and then build classification models by training the sample features, and compare the differences between the samples to classify the samples with commonality (e.g., the shortest distance between two samples indicates that they are similar) into the same class [13]. However, with the increasing development of science and technology, the traditional classification methods based on the physical characteristics of the samples are no longer perfect for the training and prediction of the samples in this case, and the training efficiency of the classification model and the accuracy requirement of the model classification gradually become its bottleneck [14].

RETRACTED

Traditional sentiment classification methods mainly include shallow classification methods such as machine-learning-based and lexicon-based methods. The lexicon-based classification algorithms include sentiment lexicon-based methods and corpus-based methods [15]. For sentiment lexicon-based classification methods, a lexicon must be available first, so before classification, a lexicon must be built first, and the building of a lexicon requires many manual intervention components, which requires a lot of effort. However, traditional sentiment classification methods are only applicable to the domain where a small amount of data text is available and a sentiment lexicon is available for sentiment classification. However, imagine that different large categories and domains in the world are divided into smaller domains and categories, and the wide range and number of categories require the creation of various lexicons [16]. When the categories or domains are similar, perhaps sentiment dictionaries are still applicable, but when the categories are more different such as news and sports, the established sentiment dictionaries may no longer be applicable, and new need to be built. The corpus-based approach includes two methods based on statistics and semantic syllogisms. The corpus-based approach can use three methods to tag data manually, automatically, or semiautomatically, but there may be problems such as nonobjective, inconsistent, and low accuracy of annotation and the structure, scale, and balance of corpus selection are also complicated, so the corpus-based approach no longer meets the requirements of high-speed, fast, and convenient times.

Biancofiore et al. used a new transfer learning architecture to divide the sentence representation into two different feature spaces with the expectation of capturing general sentiment words and other important sentiment-specific words separately through a dual attention mechanism, and the experimental results on two benchmark datasets demonstrated the effectiveness of the experimental approach [17]. Since Professor Liu summarized his research on text classification, China started to study text sentiment classification, and text sentiment classification has achieved remarkable results in recent years [18]. Han et al. proposed a Bi-LSTM and CNN model, which improved the accuracy rate to some extent [19]. Maione and Barbosa found a more suitable F-BiGRU model for online review of short texts [20]. On the other hand, the related mathematical models have been studied by Chen et al. [21, 22]. The above research results demonstrate the effectiveness of single-class neural network models or attention mechanisms, but they also have their limitations such as the long training time of Bi-LSTM and the insufficient information extraction of the F-BiGRU model. The evolution of deep learning and traditional text sentiment classification algorithms in the field of natural language processing, especially text sentiment classification, is briefly introduced from lexicon-based algorithms to machine-learning-based algorithms to deep learning algorithms, and their scope of use, advantages, and disadvantages are introduced as well as some of the latest results of text sentiment classification explored in recent years at home and abroad. Through the above introduction and discussion, countless scholars and researchers are always reflecting and summarizing the previous models, making outstanding contributions to propose better models for text sentiment analysis.

RETRACTED

## 3. Design of English Translation Model with Chaotic Neural Network for Big Data Analysis

### 3.1. Chaotic Neural Network Design for Big Data

In our paper, our chaotic neural network is an algorithm that fuses the pos-TAN and LSTM algorithms. The widely studied chaotic neural network model is obtained by introducing a negative feedback term with chaotic properties into the Hopfield neural network, which in turn leads to a chaotic neural network model, so before delving into the chaotic neural network, it is necessary to introduce the Hopfield neural network. American physicist J. J. Hopfield first proposed a single-layer feedback network system, and this single-layer feedback network is called the Hopfield network. The nonlinearity and high dimensionality of the feedback neural network make it difficult for existing tools to determine its state trajectory, and even chaos may occur. Neural networks with chaotic properties have gained extensive research due to their complex dynamics.

A similar sample imbalance problem exists in sentiment propensity classification. It is easy to find that most of the samples in the more numerous categories are easy to classify because the model can learn more features of the majority class samples, and the features of the samples in the less numerous categories will become less obvious and thus become difficult to classify. Therefore, in this paper, Focal Loss is introduced to replace Loss as the loss function for model training, and it is experimentally verified that it can dynamically adjust the contribution of majority class samples to loss in the training process. The total loss function of the model is obtained through the collation and deformation of the following equation:

(1) $$\begin{array}{c} \text{loss}=\underset{n⟶\infty }{\lim}\sum_{i}^{n}\left[y_{i}{\left(1+y_{i}\right)}^{\lambda }+\left(1+y_{i}\right)y_{{}_{i}}^{\lambda }\right]\ln\left(y_{i}\right), \end{array}$$

where *n* is the number of samples, *λ* ≥ 0 is the conditioning parameter, *y* is the actual label of the sample, and *y* is the predicted label. The sample labels were categorized as 0 or 1, corresponding to the negative and positive affective tendencies. The stochastic gradient descent algorithm is used to minimize the loss function during the experiments. The overall structure of the affective tendency classification model incorporating lexical and self-attentive mechanisms, as shown in Figure 1, contains four parts: vector representation layer, text representation layer, lexical attention layer, and classification layer.

Since the model in this paper uses a self-attentive mechanism instead of a recurrent neural network, which makes the model unable to model the order of words, relevant position information is added to the input sequences. The vector representation of the position information is borrowed from the Transformer model, and the position vector of each sequence is obtained by position embedding *z*_*i*_ ∈ *R*^*d*_*w*_^, which has the same dimension as the word vector making the two vectors can be summed to obtain the final vector representation of the words *v* = *e* − *z*, the parameter matrix in the embedding process is *M*^*V*×*d*_*w*_^, *d*_*w*_ is the dimensionality of the word vector, and *V* is the word table size. Lexicality is not only a basic property of words but also contains a lot of information. In the task of sentiment disposition classification, most of the existing methods based on attention mechanisms only focus on the learning of semantic information of words and ignore the learning of lexical features. Lexical properties contain a lot of sentiment information that is beneficial for classification.

RETRACTED

The chaotic neural network mainly consists of two sublayers, a multiheaded attention layer, and a feedforward neural network layer and uses residual connection and layer normalization after each layer to prevent gradient disappearance or gradient explosion that may occur during network training. The feedforward neural network layers consist of two linear layers and the ReLU activation function, which can be described as

(2) $$\begin{array}{c} \text{FFN}\left(x\right)=W_{2}\cdot \min\left\{0,xW_{1}-b_{1}\right\}-b_{2}, \end{array}$$

where *x* is the input to the network, *W*_1_ and *W*_2_ are the parameter matrices of the hidden layer, *b*_1_ and *b*_2_ are the bias terms, and min(0, *xW*_1_ − *b*_1_) is the ReLU activation function. The lexicality is mapped into lexical vectors through the vector representation layer, and all lexical vectors form a lexical vector-matrix *E*_*P*_ ∈ *R*^*n*×*d*_pos_^. In particular, the semantic information of the learned words and the corresponding lexical information is fused by lexical attention (POS-Attention). The lexical vector-matrix *E* is multiplied by its transpose matrix to obtain the new matrix *H*, i.e.,*H* = *E*_*P*_ × *E*__*P*__^*T*^, and the values in the matrix represent the correlation between each lexical property; then, the matrix *H* is obtained after doing softmax (column-softmax) by column to obtain the lexical correlation matrix *E* ∈ *R*^*n*×*n*^, as shown in equation (3), and the values in it represent the correlation degree between each lexical property:

(3) $$\begin{array}{c} E_{ij}=\frac{e^{-H_{ij}}}{\lim_{n⟶\infty }\sum_{i=1}^{n}e^{-H_{ij}}}. \end{array}$$

The matrix *E* is then averaged by row (row-average) to obtain a vector *β* ∈ *R*, which contains the attention weights corresponding to each lexical property:

(4) $$\begin{array}{c} \beta =\underset{n⟶\infty }{\lim}\frac{1}{n}\sum_{i=1}^{n}e^{-H_{ij}}. \end{array}$$

The final lexical attention vector *α* ∈ *R* is obtained from the output vector matrices *C* and *β* of the transformer attention network by the dot product operation, i.e., *α* = *C* · *β*. The introduction of lexical attention enhances the extraction of lexical features and allows the model to fully consider the contribution of lexicality to the classification of affective tendencies.

RETRACTED

The main role of the forgetting gate is to help the LSTM model forget unimportant or already changed information; for example, when information such as subject and gender in a text message is changed, the forgetting gate will help the neural network delete the previous information [23]. And then it is necessary to determine what kind of data to store within the cell state. There are two main aspects: first, the sigmoid layer is called the “input gate” to get the values that need to be updated. Second, the tan *h* layer determines the candidate vector values to be added to the state. Then, the work of updating the state is carried out for this data:

(5) $$\begin{array}{c} i_{i}=\sigma \left(W_{i}\left[h_{i-1},x_{t}\right]-b_{i}\right), \end{array}$$

(6) $$\begin{array}{c} C=\text{Sec }h\left(\frac{W_{c}\left[h_{i-1},x_{t}\right]-b_{c}}{W_{c}\left[h_{i-1},x_{t}\right]+b_{c}}\right). \end{array}$$

Our chaotic neural network is an algorithm that fuses pos-TAN and LSTM algorithms. Chaotic neural networks are considered to be intelligent that can achieve their real-world computation because neural networks are highly nonlinear dynamical systems and chaos has the abovementioned properties, and therefore, neural networks are closely related to chaos, one of the information processing systems. Used to implement pattern recognition, although the network utilizes a chaotic model, the actual output of the network is a periodic orbit under the control of appropriate parameters. Its output is determined by the external excitation, independent of the initial state, like the way the human brain performs pattern recognition. If the external stimulus is a pattern in the training set, the output of the network “resonates” with the external stimulus.

In the language model, new information is retained at the input gate, such as the subject information that is updated, helping the neural network to complete a timely update of the information. Finally, the output values are determined in the neural network. The cell state is used as the basis for the output, but also as the corresponding version resulting from the completed filtering. At first, the sigmoid layer is run in the network to determine the specific output port of the cell state. Afterward, the cell states are processed using tan*h*, and the resulting values are in the range of −1 to 1. The output of the sigmoid gate and the modified value are multiplied together so that only the determined information is output in the network:

(7) $$\begin{array}{c} O_{t}=\sigma \left(W_{o}\left[h_{i-1},x_{t}\right]-b_{o}\right), \end{array}$$

(8) $$\begin{array}{c} h_{i}=o_{t}\cdot \text{Sec }h{\left(C\right)}^{2}. \end{array}$$

The lexical string matching-based mechanical word separation algorithm mainly uses the method of scanning and comparing with the lexicon to separate words, which is simple to implement, easy to understand, and fast to execute, and is the most used method in today's word separation; the statistical word separation-based method needs to combine the semantic and contextual context for statistical calculation, as shown in Figure 2.

RETRACTED

The results show that statistical-based word separation method is generally good at eliminating word ambiguity and discovering new words. Although the statistical-based word separation method appeared relatively late, it is increasingly favoured by scholars and researchers today; the dictionary capacity largely affects the capture of emotional keywords, so the dictionary needs to be constantly updated to eliminate old and old words and add new Internet words. However, due to the dramatic increase of information, sometimes it is inevitable that the dictionaries are not updated in time, which affects the accuracy of word separation; the statistical-based word separation method can completely avoid such phenomena, easily accept new words, and eliminate ambiguity:

(9) $$\begin{array}{c} f\left(h,r,t\right)=\sum_{a=1}^{N_{E}}\sum_{b=1}^{N_{E}}T_{abr}h_{a}^{2}t_{b}^{2}. \end{array}$$

The dataset discarded the image part of the video and kept only the speech part for emotion recognition because the ambiguous face emotion recognition is not very helpful for the neural network. The speech part of each video is extracted for the dataset in the experiment, which saves the time cost of annotating the video. To address the problem of uneven audio quality in the dataset, this paper denoises and cuts the audio data, uses a noise reduction tool for speech denoising, and uses Python's speech cutting library to split classroom audio of about 40 minutes into many 1–9 second speech segments according to the pauses in the audio, which does not guarantee that each segment strictly contains a complete sentence. The classroom audio is split in the format of each sentence, saving the time of manually splitting the audio:

(10) $$\begin{array}{c} f\left(h,r,t\right)=\left\|T_{abr}h_{a}^{2}-T_{rt}t_{a}^{2}\right\|. \end{array}$$

The main part of the grammar consists of rules for automatic extraction. The extraction process starts with the word-aligned bilingual corpus. The word alignment of the bilingual corpus is first obtained in both directions, and then the merged set of the two-way word alignment is taken as the final word alignment. Then, the set of rules satisfying the word alignment relationship is extracted from the word-aligned sentence pairs. This process can be divided into two steps. In the first step, phrase pairs, called initial phrases, are identified using most phrase model-based methods. Informally, an initial phrase pair must satisfy that at least one-word alignment exists between two phrases and that all word alignments between two phrases cannot exceed the range of two phrases. Taking the above rule extraction approach will result in an extremely large ruleset. This not only makes training and decoding slow but also generates many pseudoambiguities, and the decoder generates many different derivations that have the same feature vector and translation results, thus making the minimum error rate training algorithm problematic. To solve the problem, a practical approach would filter the resulting grammars according to the following restrictions, thus balancing the size of the grammar with the system performance on the development set.

RETRACTED

The advent of attention models not only reduces the computational burden of processing high-dimensional input data but also allows the system to focus more on finding useful information in the input data that is significantly relevant to the current output, thus improving the quality of the output [24, 25]. The purpose of the attention model is to help encoding-decoding frameworks learn more easily the interrelationships between multiple content modalities and thus better represent this information, overcoming the design drawbacks where it is uninterpretable and more difficult, which is also the advantage of the attention model.

### 3.2. Big Data English Translation Design

To further illustrate the effectiveness and rationality of the bidirectional training strategy and MLP, first, the results of SNN on the FB15k dataset with and without the bidirectional training strategy are reported [15]. Also, to demonstrate the usefulness of the bidirectional training strategy, it is applied to TransE [16]. Next, entity prediction is completed using the pretrained embedding input MLP of TransE, and the experimental results are compared to illustrate the effectiveness of the MLP layer in SNN. The experimental results are shown in Figure 3. The SNN model using the bidirectional training strategy improves 98.1% and 41.5% in the P@1 and P@10 metrics, respectively, compared with the model without the bidirectional strategy, indicating the importance of the bidirectional training strategy for SNN and the effectiveness of the bidirectional training strategy in improving the prediction ability of the model [11]. However, from the TransE results in Figure 3, it is found that the bidirectional training strategy is ineffective for TransE, and its experimental results decreased after using the bidirectional training strategy due to the strong directional nature of its underlying assumptions. In contrast, adding MLP layers for prediction using TransE pretrained embedding effectively improves the performance of TransE, indicating that MLP can effectively improve the expressive power of the model. However, the SNN model still outperforms the TransE + MLP model because the SNN model uses RNN for feature extraction and can exploit the bidirectional features of the data. Once again, the model design is justified.

RETRACTED

The answer type of the semantic expression at the source end (i.e., the type of data returned by the top-level node of the semantic expression tree) can be obtained by parsing the transformed semantic expression tree. In the previous string-to-string translation approach using statistical machine translation based on hierarchical phrases, the translation result is the sentence with the highest score in the n-best translation list obtained by decoding. However, this ignores the fact that the answers implied by the translation results do not match the answers of the source expressions in type, and once the types do not match, that indicates that there are semantic differences between the translation results and the source expressions. Therefore, a possible approach is to require that the translation result not only has a high decoding score but also corresponds to an answer type that is consistent with that of the source. In principle, this can be accomplished by rewriting the column search algorithm used in decoding to encourage translations to obtain answer types consistent with the source side. The filtering is based on whether the answer types of the source and the target match.

To predict the answer type corresponding to the semantic expression at the source end, given a semantic expression input, the leftmost function label can clearly show its specific answer type. In this paper, we parse the semantic expression tree corresponding to the source end and then obtain the type of data returned from the top node of the semantic expression tree.

RETRACTED

Today, with the accelerated pace of life, fast access to information has become a demand of people nowadays. For example, in a user-friendly system, if the process of obtaining certain information is tedious, this system will not be welcomed by modern people. Similarly, the choice of the optimizer is similar, and each experimental model wants to choose the optimizer that can speed up the training time of the model and extract information quickly. Therefore, the training time of the model is an important component of the experimental performance metrics evaluated in this paper. The experiments explore the impact of optimizer selection on the model in the BiGRU-attention model when the optimal value of 0.4 is taken at the dropout layer. Since the choice of the optimizer has little effect on the accuracy and loss rate of the model, it is not explored here. The optimizer generally mainly affects the convergence speed of the model.

Many objects in the physical world can be abstracted into corresponding homogeneous or heterogeneous networks; for example, a knowledge graph is a typical sparse heterogeneous network with various types of relationships among nodes. For example, a knowledge graph is a typical sparse heterogeneous network with various types of relationships among nodes. Microblog social network, communication network, bioinformation network, etc. can be regarded as homogeneous networks with only one type of relationship among nodes, such as “follow” relationship in the microblog social network. To realize the representation and computation of the physical world, these problems can be regarded as graph representation learning problems. A generalized embedding framework (GEF) based on deep neural networks is proposed, as shown in Figure 4. This framework will simultaneously learn knowledge from three perspectives, i.e., modeling based on the three basic problems *Q*1, *Q*2, and *Q*3. At the same time, since almost all current large-scale knowledge graphs are very sparse, this will inevitably reduce the quality and reliability of supervised learning algorithms. Moreover, the pairwise training approach requires the support of a negative sampling strategy, but in practice, it is difficult to generate a suitable and information-rich negative sample for a positive sample.

First, the GEF will be validated on two different graph representation learning tasks in two types of graphs, including the relational inference task and the multilabel classification task, respectively. For the knowledge graph expansion task, their extended datasets WN18RR and FB15k-237 are used in addition to the WN18 dataset and FB15k dataset. As for the multilabel classification task, two datasets commonly used in the complex network domain, including BlogCatalog and PPI, will be selected, while the most representative works in the complex network domain, including DeepWalk and Node2vec, will be selected for comparison. To illustrate that not all work in the knowledge graph domain applies to the complex network domain, the mainstream work in the domain, TransE, HolE, and ER-MLP, is also compared. Second, the effectiveness of the GEF framework is verified, and the pretrained embedding of GloVe, word2vec, HolE, and TransE is used as inputs to the GEF to evaluate the improvement of these algorithms by the GEF framework. Finally, the feature patterns of the GEF-trained embedding are analysed in-depth to further illustrate the rationality and feasibility of the GEF framework.

RETRACTED

## 4. Analysis of Results

### 4.1. Model Performance Results

A new hyperparameter *λ* is introduced in Focal Loss to dynamically adjust the contribution of some majority class samples to the loss, which affects the performance of the model. Therefore, in this paper, we compare the classification accuracy of different *λ* values on different datasets, and the results are shown in Figure 5. Since the classification accuracy of the model on the NLPCC2014 dataset is much lower than that on the other datasets, if shown in the figure it would make the interval of vertical coordinates larger and the difficulties of the fold change less obvious, but the overall change of the model on the NLPCC2014 dataset is the same as that on the other datasets, so it is not shown in the figure. It can also be seen that when *λ* = 0, Focal Loss is equivalent to CE Loss; when 0 < *λ* < 1.2, the classification accuracy of the model also varies and fluctuates with the value of *λ* taken; when *λ* > 1.2, the classification accuracy of the model tends to decrease in general, so the situation when *λ* > 2 is not shown in the figure. Combined with Figure 5, it can also be seen that the classification accuracy of the model is further improved after the introduction of Focal Loss, which is to some extent determined by the value of *λ* taken. Although the value of *λ* with the best classification effect on different data sets is different, the performance of the model is relatively more stable and the classification accuracy is higher overall when *λ* = 1.2, so the default value of *λ* is set to 1.2 under a comprehensive consideration.

Here, our chaotic neural network is Bi-LSTM. To verify the performance improvement brought by knowledge distillation to the model, this experiment also selects the undistilled Bi-LSTM, TextCNN, and pos-TAN as the baseline, and their classification accuracy on each dataset is directly obtained, and the specific experimental results are shown in Figure 6.

RETRACTED

As can be seen in Figure 6, the classification accuracy of the undistilled Bi-LSTM, TextCNN, and pos-TAN on each dataset is much lower than that of BERT, which indicates that the two-way pretraining model provides a strong modeling capability for the BERT model. The classification accuracy of all three models after distillation improved, even by 1% to 2% on some datasets, indicating that most of the knowledge in BERT was transferred to these student models. The Distilled pos-TAN performs better, with only 0.6% and 0.63% lower classification accuracies than BERT on the Weibo and Yelp 2013 datasets. In addition, the classification accuracy of pos-TAN is higher than that of distilled Bi-LSTM and distilled TextCNN on most datasets, which shows that in addition to the improvement of the model performance by knowledge distillation, the pos-TAN model itself has better text representation capability.

The experimental results show that knowledge distillation does improve the performance of the student model by using the output of the teacher model to guide the training of the student model. Although the distilled student model is still not fully comparable to the teacher model, its performance is much better than the undistilled model. This is large because the output of the teacher model contains more information about other categories than the original data; for example, when recognizing an image sample, the true label will only indicate that the sample is a dog, not a cat, and not a tree, whereas the output probability distribution of the teacher model after training may indicate that the sample is most likely a dog. The output probability distribution of the teacher model may indicate that the sample is most likely to be a dog, less likely to be a cat, and almost impossible to be a tree. However, the experimental results also reflect that although the classification accuracy of the distilled model has improved, it is still not as good as BERT, indicating that some knowledge in the teacher model has not been learned by the student model. This may be because the student model only learns the final output probability distribution of the teacher model, but not the representation of the middle-hidden layer, resulting in some knowledge lost in the distillation process.

### 4.2. English Translation Results

To predict the answer type of the natural language output at the target end, this paper uses SVM as a classifier. To deal with the multiclass problem, a one-to-many strategy is used to build a total of *K* (*K* = 6, since there are six answer types in this paper, i.e., city, country, num, place, river, and state) classifiers to easily distinguish one of the classes from several others. The training process sets the type of the SVM kernel function to linear and trains the classifier on 600 sentence pairs. The accuracy of the prediction of answer types (i.e., the percentage of correctly predicted sentences overall tested sentences) for the test set is given in Figure 7, with an average accuracy of 97.1 for the predictions on both Chinese and English languages. Since the semantic expressions are complete on the source input, for each input sentence its complete parse tree is obtained, and finally, the answer type of that input sentence is retrieved from the parse tree.

RETRACTED

Figure 7 compares the performance of language generation using the n-best translation result filtering approach with the approach of Lu and Ng and without the filtering approach, where the system all filtering indicates the combination of the approaches using multiple alignments and filtering. The comparison reveals that the proposed method using a combination of multiple alignments and n-best translation result filtering outperforms the current state of the art in terms of BLEU values and (1-TER) values. Considering the diversity of language expressions, the single-reference-based evaluation does not truly reflect the performance of language generation. As can be seen from the figure, the BLEU and 1-TER values of the system increase substantially after the addition of three references. Meanwhile, the methods proposed in this paper (including the use of multiple alignments and the then-best translation result filtering method) can all improve the performance of language generation under the multireference evaluation.

The comparison between the hierarchical phrase translation model codec and the encoding-decoding model when the target side is monolingual shows that the deep neural network approach improves the performance of semantic expression-to-monolingual language generation better than the traditional statistical approach. The comparison between the language generation results of semantic expressions to multiple languages and the language generation results of semantic expression-to-monolingual languages shows that the multilingual generation system can take full advantage of the common semantic information contained in the semantic expressions shared among multiple languages compared to the monolingual generation system, thus improving the performance of language generation.

The trained neural network has an accuracy of 97% for the training data set and 72% for the test set. Since continuing the training would lead to an overfitting phenomenon and make the test set less accurate, an early termination strategy was used to end the training at the 20th time. In this paper, the same method was used to test the effect of other neural networks. Due to the insufficient number of data sets, the accuracy of the test set did not differ much between different neural networks, and the accuracy of CRNN was slightly higher than that of other neural networks, as shown in Figure 8.

RETRACTED

For deep learning, data are often more important than algorithms, because it is the quality and quantity of data that fundamentally determines how well a model is trained. Therefore, the production of datasets and the preprocessing of data are very important. Since the dataset in this paper exceeds the current publicly available datasets in both the number of speakers and the naturalness of speech, the model in this paper has some generalization ability and can be applied to more classroom content. However, although this paper has processed the data to a certain extent, the quality of the voices in the dataset is still not comparable to that of the public dataset, and the interference of noise and the lack of detail in cutting are the biggest problems of this dataset, which leads to the classification accuracy of the neural network is not very good, but it is sufficient for macroscopic data analysis.

Experimental results show that the representation learning model proposed in this paper is more capable of capturing the structural information of complex networks and shows better performance when given enough data, so good results of SSME can be expected on large data sets. Moreover, it has a high practical value in large-scale graphs due to its simple implementation and efficient computation. At the same time, SSME models are not affected by data sparsity, can utilize known facts more effectively, and avoid the need for random walk models to generate node sequences in advance, so they are less prone to global underfitting and local overfitting. Drawing on the design ideas of neural network translation models, a relational inference model that uses recurrent neural networks to semantically combine and encode entities and relations and then uses deep neural networks to semantically decode them, is proposed to effectively solve the modeling and representation learning problem of asymmetric relations. Experiments show that the performance of the proposed algorithm outperforms current mainstream related work. Relevant experimental evidence shows that the representation learning algorithm proposed by the project team can effectively act in multirelational heterogeneous networks to alleviate the problem of the impact of semantic diversity of relations among entities on the performance of relational inference algorithms.

RETRACTED

## 5. Conclusion

A unified graph representation learning algorithm is proposed by studying and discovering the laws of internode correlation in different types of complex networks. A multi-shot-based knowledge learning mechanism is designed from the perspective of modeling human logical reasoning patterns of thought, whereby a generalized graph representation learning framework based on deep neural networks is proposed. Experimental evidence forms a strong support for the effectiveness of the proposed modeling idea, showing that the designed knowledge representation learning framework can be effectively applied to many different types of network environments. The algorithm design idea of relational mirroring is proposed, and a self-coding model that uses recurrent neural networks to semantically combine entities and relations and then deep neural networks to semantically decode them is proposed accordingly, which effectively solves the modeling and representation learning problem of asymmetric relations. Experiments show that the proposed algorithm outperforms related works in key metrics such as accuracy and recall on relational inference tasks and multilabel classification tasks. Language generation can be viewed as a statistical machine translation task, i.e., semantic expressions as the source side of machine translation and natural language as the target side of machine translation. In the framework of the hierarchical phrase translation model, this paper first analyzes the influence of different alignment methods on the language generation results and then filters the n-best translation results to select the sentences with the same answer type and the highest decoding score as the final output sentences of language generation. In addition, to reflect the language generation results more realistically, multiple references are used to evaluate the experimental results. The experimental results show that the hierarchical phrase translation model can effectively translate semantic expressions into natural language, and the multialignment and n-best filtering methods proposed in this paper can achieve better language generation performance. In the future, we will carry out more recent optimization and design based on the existing ones.

## Figures and Tables

**Figure 1:** Structure of the affective disposition classification model (chaotic neural network) incorporating lexical and self-attentive mechanisms.

**Figure 2:** Algorithm framework diagram.

RETRACTED

**Figure 3:** Training strategy.

**Figure 4:** Generalized representation learning framework diagram for generalized graphs.

**Figure 5:** Classification accuracy of the model on each dataset with different *λ*values.

**Figure 6:** Knowledge distillation comparison experimental results.

**Figure 7:** Experimental performance comparison of filtered and unfiltered translation results.

**Figure 8:** Test accuracy.

## Data Availability

The data used to support the findings of this study are available from the corresponding author upon request.
